The article "Construction of an Immune-Autophagy Prognostic Model Based on ssGSEA Immune Scoring Algorithm Analysis and Prognostic Value Exploration of the Immune-Autophagy Gene in Endometrial Carcinoma (EC) Based on Bioinformatics" was retracted in 2023. Reasons: signs of a paper mill; suspected computer-generated content; unreliable results or conclusions; concerns about the data.

# Construction of an Immune-Autophagy Prognostic Model Based on ssGSEA Immune Scoring Algorithm Analysis and Prognostic Value Exploration of the Immune-Autophagy Gene in Endometrial Carcinoma (EC) Based on Bioinformatics

**DOI:** 10.1155/2022/7832618

**Published:** 2022-02-22

**Authors:** Xiaomin Xu, Fang Lu, Cheng Fang, Shumin Liu

**Affiliations:** ^1^Heilongjiang University of Chinese Medicine, Harbin, China; ^2^School of Continuing Education, Heilongjiang University of Traditional Chinese Medicine, Harbin, China; ^3^Drug Safety Evaluation Center of Heilongjiang University of Traditional Chinese Medicine, Harbin, China

## Abstract

**Background:**

Endometrial carcinoma (EC) is a malignant cancer spreading worldwide and in the fourth position among all other types of cancer in women. The purpose of this paper is to explore the prognostic value of the immune-autophagy gene in endometrial carcinoma (EC) based on bioinformatics, construct an immune-autophagy prognostic model of endometrial carcinoma, search for independent prognostic markers, and finally predict the potential therapeutic drugs of TCGA subgroup.

**Methods:**

The Cancer Genome Atlas (TCGA) database was used to extract transcriptome sequencing data of patients suffering from EC; 28 kinds of immune cells were scored by ssGSEA, and the immune subtypes were grouped by consistency cluster analysis. The accuracy and effectiveness of the grouping were verified by the analysis of differential gene expression and survival rate of immune checkpoints in the two groups to provide the premise and basis for the establishment of independent prognostic factors. The expression of different genes in high and low immune groups was analyzed. The analysis of various genes' expression in immune groups (high and low) has been performed. Go function annotation and KEGG pathway enrichment analysis were used to evaluate the difference of immune infiltration between high and low immune groups. The immune and autophagy genes were crossed, the key (hub) genes were selected, the risk was scored, the prognosis model was constructed, and the independent prognostic markers were established. CAMP and CTRP 2.0 were used to test the drug sensitivity.

**Results:**

According to the level of immune cell enrichment, the results have been subcategorized into two immune subtypes: high immunity group_ H and low immunity group_ L. Two immune subtypes, CD274, PDCD1, and CTLA4, were detected in the immune system_ H and immunity_L. A significant difference was detected between these two groups in the expression and survival rate. Few more differences were also detected between the two groups through the evaluation of immune infiltration, which proved the grouping's accuracy and effectiveness. Differential gene expression analysis showed that there were 721 DEGs and 3 hub genes. DEGs are mainly involved in lymphocyte activation, proliferation, differentiation, leukocyte proliferation, and other biological processes, mediate chemokines' activities, chemokine receptor binding, and other molecular functions, and are enriched in the outer plasma membrane, endoplasmic reticulum, and T cell receptor complex. The enriched pathways are allograft, complex, inflammatory, interferon-alpha, interferon-gamma, E2F, G2M, mitotic, etc.

The article "Construction of an Immune-Autophagy Prognostic Model Based on ssGSEA Immune Scoring Algorithm Analysis and Prognostic Value Exploration of the Immune-Autophagy Gene in Endometrial Carcinoma (EC) Based on Bioinformatics" was retracted in 2023. Reasons: signs of a paper mill; suspected computer-generated content; unreliable results or conclusions; concerns about the data.

**Conclusion:**

Through bioinformatics analysis, we successfully constructed the immuno-autophagy prognosis model of endometrial cancer and identified three high-risk immunoautophagy genes, including VEGFA, CCL2, and Ifng. Four potential therapeutic drugs were predicted as sildenafil, sunitinib, TPCA-1, and etoposide.

## 1. Introduction

Endometrial carcinoma (EC) is a tumour of epithelial cells that arises from the endometrium, which is the most prevalent gynaecological malignant tumour and on the fourth position among all other types of cancers in women worldwide [1]. According to available statistics data, about 140000 women worldwide are diagnosed with endometrial cancer per year, with an estimated 40000 women dying due to this disease. The standard endometrial cancer age curve indicates that most cases are discovered after menopause, with the largest prevalence rate occurring in the seventh ten years of life [2].

In the last decades, the incidence rate of EC has been increasing worldwide. In recent times, based on clinical manifestations, timely diagnosis of EC patients can be made; these manifestations include postmenopausal bleeding and tumour markers' abnormal levels [3]. At the same time, about 15% of EC occurs in women with no vaginal bleeding [4]. For example, various serologic markers in EC diagnosis, a carbohydrate antigen 19-9, and carbohydrate antigen-125 were identified, but only in 20%, −30% of EC patients were under control [5]. Because of late diagnosis, EC patients cannot be adequately treated, resulting in more risk of metastatic cancer and poor prognosis [6, 7]. Despite the progress of treatment methods, the prognosis of advanced endometrial cancer is still a big challenge. Therefore, this study aims to build a prognostic model of EC and find more reliable and accurate prognostic biomarkers so that the EC patient's survival rate can be improved.

Much evidence shows that tumour immune cell infiltration is very much similar to the occurrence and development of cancer [8–10]. In tumours, the type and proportion of immune cell infiltration are closely related to clinical results, which have predictive value for patients' survival and can affect the therapeutic effect of the tumour, so it is expected to become a drug target and clinical biomarker [11, 12]. The neutrophils associated with tumours are the main types of immune cells, which can eliminate the growth of pathogens and prevent host from microbial infection and are associated with breast cancer and gastric cancer prognosis [13–15]. Besides, tumour-associated macrophages are involved in EC's invasive progression [16, 17]. Simultaneously, some studies have shown that the induction of autophagy is very much similar to the poor prognosis of endometrial cancer [18]. Autophagy involves the survival, differentiation, metabolism, immunity, and other physiological functions of normal cells and tumour cells. The relationship between autophagy and cellular immunity has attracted more and more attention. There are still many problems in EC autophagy studies: first, most of the current research limitations and stromal and epithelial cells; very little research on immune cells and endometrial stem cells. Secondly, in many studies, the sample size is small. The detection of autophagy pairs is not comprehensive enough to be limited to detecting partial autophagy-related protein or RNA levels that do not represent dynamically varying autophagy levels. Thus, this study will construct the prognostic model based on immune-autophagy. The prognostic model based on immune-autophagy has the following advantages: (1) supplementing the EC research at the immune cell level; (2) making the prognosis model more stable and effective; (3) compensating for the limitations of single autophagy; and (4) providing the corresponding foundation for exploring the relationship between tumour cell autophagy and cell immunity to lay the foundation for the further study of EC.

The article "Construction of an Immune-Autophagy Prognostic Model Based on ssGSEA Immune Scoring Algorithm Analysis and Prognostic Value Exploration of the Immune-Autophagy Gene in Endometrial Carcinoma (EC) Based on Bioinformatics" was retracted in 2023. Reasons: signs of a paper mill; suspected computer-generated content; unreliable results or conclusions; concerns about the data.

## 2. Materials and Methods

### 2.1. Identification of EC Subtypes Based on Immunocyte Transcriptome

The TCGA knowledge base was used to download the gene expression data of 536 patients having EC. Each EC data set has been classified using 28 immune cell gene sets. Then, mRNAseq of normalized RSEM/RPKM value with log2 was transformed as the input RNAseq data for the clustering. RSEM is used to estimate gene and transcript abundances and these values are normalized to a fixed upper quartile value of 1000 for gene and 300 for transcript level estimates. RPKM for a given GeneX is calculated by (raw read counts ^*∗*^ 10^9)/(total reads ^*∗*^ length of GeneX). Total reads are the lane yield after removing poor quality reads and the length of GeneX is defined as the median length of all transcripts associated with GeneX. The R language GSVA, Lima, GSEABase software package was used to perform analysis known as ssGSEA [19], and 28 kinds of immune cells were scored [20, 21] to quantify the enrichment level of gene set in each EC sample. According to the enrichment degree of immune cells, they have been classified into high immunity group and low immunity group. To quantify the gene set in each EC sample, the software package Consensus Cluster Plus was used for the consistency cluster analysis of the ssGSEA score. The estimate package was used to draw the heat map and predict the purity of the tumour. The optimal clustering number is determined by the clustering score of the CDF curve.

### 2.2. Immune Checkpoints in Different EC Subtypes in Immunotherapy

PDCD1, CTLA4, and CD274, three immune checkpoints, are closely related to multiple types of tumour prognosis [22–24]. At the same time, the high expression of immune checkpoints PDCD1, CTLA-4, and CD274 is associated with the prolongation of the overall survival of tumour patients. Therefore, we studied the PDCD1, CTLA4, and CD274 expression in each subtype. Subsequently, the survival rate difference analysis of immune checkpoint inhibitor treatment was used to verify.

### 2.3. Survival Verification and Difference Analysis

The survival, surviving software package is used to analyze the difference in survival rate. The differences have been described using the Kaplan–Meier curve in EC patients and their survival rates in multiple classified immune cell subtypes datasets. The survival outcomes of EC patients compared to detect the difference in survival time was significant. The differences between the two subtypes were analyzed. DEGs meet the requirements of *P* < 0.05 and FC <1.5 and draw the related volcanic map and thermal map to visually show DEGs' differential expression.

### 2.4. Enrichment Analysis of DEGs Gene and Evaluation of Immune Infiltration Degree

#### 2.4.1. Functional Enrichment Analysis of DEGs Gene

After processing the TCGA data, it is divided into two subtypes using consistent clustering analysis. The two subtypes of immunity_H and immunity_L are analyzed for related differences, and Limma is used for differential expression analysis and output DEGs and to draw the corresponding volcano map and heat map [25]. The functional enrichment analysis of immunological differentially expressed genes is performed. GO functional annotation covers all biological processes. To analyze the function of DEGs, the cluster profile package of R software was used to annotate the go function of DEGs and analyze the enrichment of the KEGG pathway. GSEA analyzed KEGG; the cut-off standard was set as FDR <0.05 and *P* < 1.5, and the analysis results were visualized.

The article "Construction of an Immune-Autophagy Prognostic Model Based on ssGSEA Immune Scoring Algorithm Analysis and Prognostic Value Exploration of the Immune-Autophagy Gene in Endometrial Carcinoma (EC) Based on Bioinformatics" was retracted in 2023. Reasons: signs of a paper mill; suspected computer-generated content; unreliable results or conclusions; concerns about the data.

#### 2.4.2. Immune Infiltration Evaluation

The CIBERSORT [26] was used to analyze the immune infiltration of 22 kinds of immune cells. Through the analysis, it can still be concluded that there are differences in immune infiltration between groups.

#### 2.4.3. Screening of Key (Hub) Genes and Construction of Prognosis Model

The list of related genes was downloaded from the autophagy database and immune database. Immune genes (import), autophagy genes (HADB), and differentially expressed genes (DEGs) were drawn by Venn map to get the essential genes. The obtained hub was analyzed by single factor Cox regression analysis. Forest map was drawn by the R package to show its expression in different subtypes and then screen the genes related to the prognosis of endometrial cancer. At the same time, the ggrisk package was used to group test the hub further to evaluate the rationality and accuracy of the prognosis model.

#### 2.4.4. Drug Sensitivity Test

The drug sensitivity data of CCLE are derived from the cancer therapeutics response portal and PRISM replicas datasets. Both datasets provide the area under the dose-response curve as a measure of drug sensitivity. The lower the AUC value, the higher the sensitivity to treatment [27]. The Camp database [28] uses gene expression characteristics to predict small molecular compounds for specific diseases. The up- and downregulation genes were uploaded to the query page in Camp, and small molecule drugs that might treat EC were searched. The range from −1-1 scores represents the correlation between the drug and the DEG. A drug with more negative correlations indicates a more significant correlation with uploaded DEG.

### 2.5. Analysis of Results

#### 2.5.1. Identification of EC Subtypes Based on Immune Cell Genome

Each sample of tumour was divided into *K* (*k* = 2–10) subtypes using the Consensus Cluster Plus software package. PAC algorithm verifies that when *k* = 2, the CDF curve provides the best segmentation, as shown in Figure 1(b). In addition, the analysis results represented that the ssGSEA scores based on 28 immune cell gene sets were divided into two subtypes, as shown in Figures 1(a)–1(f). They were defined as high immunity group and low immunity group, divided into 264 immunity_ H and 272 immunity_ L. At the same time, the comparison of matrix content showed the same trend (immunity_ H＞immunity_ L _ H＜immunity_ 50), as shown in Figure 1(g). Therefore, it can be verified that the classification of immune subtypes is accurate and reasonable.

#### 2.5.2. The Therapeutic Effect of Immune Checkpoint Inhibitors in Different EC Subtypes

The immunotherapy was observed by screening CD274, PDCD1, CTLA4, and other genes. The immunotherapy of PDCD1, CTLA-4, and CD274 was observed in immunity_ H, and immunity_ L expression was analyzed, as shown in Figures 1(d)–1(f). It was found that it was all in the immunity_. The high expression of *h* was significant (*P* < 0.05). It is suggested that the above genes have an immunotherapeutic effect and sensitivity to the treatment of immunosuppressants. At the same time, its differential expression in the immunity_H and immunity_L groups also verified the reliability and stability of the grouping.

The article "Construction of an Immune-Autophagy Prognostic Model Based on ssGSEA Immune Scoring Algorithm Analysis and Prognostic Value Exploration of the Immune-Autophagy Gene in Endometrial Carcinoma (EC) Based on Bioinformatics" was retracted in 2023. Reasons: signs of a paper mill; suspected computer-generated content; unreliable results or conclusions; concerns about the data.

#### 2.5.3. Survival Verification and Difference Analysis

The survival rate difference analysis of immunity_H and immunity_L showed that *P*=0.05 was significant, as shown in Figure 2(a). The difference between the two groups of immune genes was analyzed, DEGs met *P* < 0.05 and FC <1.5, and related volcano maps and heat maps were drawn, as shown in Figures 2(b) and 2(c). Among them, there were 721 GEGs genes, 633 genes upregulated, and 88 genes downregulated.

#### 2.5.4. DEGs Gene Enrichment Analysis and Immune Infiltration

The GO and KEGG signalling pathways of the 721 differentially expressed genes were analysed. The upregulated DEG genes were mainly related to the allograft (allograft inflammatory factors), complement (complement system), inflammatory (inflammatory mediators), interferon-alpha (INF-*α*), and interferon-gamma (IFN-*γ*) pathways; the downregulated DEG genes were mainly related to E2F, G2/M, mitotic (spindle mitosis), and other pathways, as shown in Figures 3(a)–3(b). They were mainly involved in the biological processes of lymphocyte activation, proliferation, differentiation, and leukocyte proliferation, and they mediated chemokine activities and the binding of chemokine receptors. They were enriched in the plasma membrane's outer part, endoplasmic reticulum, and T cell receptor complex, as shown in Figure 3(c). Meanwhile, the immunoinfiltration analysis showed that there was a difference in immune infiltration among the groups. The immune score of the high immune group was higher than that of the low immune group. M1 macrophages, M0 macrophages, CD8 T cells, M2 macrophages, dormant memory CD4 T cells, activated NK cells, monocytes, dormant dendritic cells, and follicular helper T cells were significantly higher in the high immune group than those in the low immune group, as shown in Figure 3(d).

#### 2.5.5. Selection of Hub Gene, Construction, and Evaluation of Prognosis Model

By using the Human Autophagy Database (HADB) and immune database (import, https:0//www.immport.org/) to download the list of related genes, draw Venn map of immune genes, autophagy genes, and 721 differentially expressed genes and find that there are three overlapping genes, such as (Figure 4(a)) VEGFA, CCL2, and Ifng, in which VEGFA is upregulated and CCL2 and Ifng are downregulated. Based on the single factor Cox regression analysis, the prognosis-related immune and autophagy genes were determined, and the prognosis models of immunity and autophagy were constructed. A risk curve was drawn for the grouping (Figure 4(b)) to further evaluate the prognosis model's predictive ability. The risk curve represented that the independent prognosis analysis of Cox was performed, and the forest map is drawn in Figure 3(d).

The article "Construction of an Immune-Autophagy Prognostic Model Based on ssGSEA Immune Scoring Algorithm Analysis and Prognostic Value Exploration of the Immune-Autophagy Gene in Endometrial Carcinoma (EC) Based on Bioinformatics" was retracted in 2023. Reasons: signs of a paper mill; suspected computer-generated content; unreliable results or conclusions; concerns about the data.

The results showed that in the single factor independent prognosis analysis, the risk score *P* < 0.05, indicating that the risk score could be used as an independent prognostic molecule; VEGF, CCL2, and IFN were all *P* < 0.05, indicating that the above genes could be used as independent prognostic factors. Also, the three genes of VEGF, CCL2, and IFN were tested by ggrisk, such as Figure 4(d), and we found that the three genes had a better classification effect, indicating that the constructed prognosis model was accurate.

#### 2.5.6. Drug Sensitivity Test

The 150 upregulated genes and 88 downregulated genes were selected and imported into CMAP to obtain the drug table; Venn intersected two drug sensitivity database data of CTRP 2.0, as shown in Figure 5(a); Spearman correlation analysis and differential drug response analysis were performed for 19 compounds, as shown in Figures 5(b) and 5(c). The lower the value on the *Y*-axis of the box graph, the higher the drug sensitivity. Results: four kinds of susceptible drugs sildenafil, sunitinib, TPCA-1, and etoposide were obtained. Relevant studies have shown that sildenafil, a phosphodiesterase 5 (PDE5) inhibitor, can activate cGMP signal transduction in mouse colonic mucosa, resist barrier dysfunction induced by DSS (dextran sodium sulfate), reduce bone marrow cell infiltration, and reduce the expression of iNOS, IFN-*γ* and IL-6, thus effectively inhibiting inflammation-driven colorectal cancer in mice [29]. Sunitinib, a tyrosine kinase inhibitor (TKI), can inhibit the migration and invasion of RCC cells by reducing the expression of mir-452-5p [30, 31]. Topoisomerase II inhibitor etoposide has been successfully and widely used to treat various types of cancer in children and adults [32].

## 3. Discussion

In this study, the bioinformatics analysis method was used to search for the relevant data of endometrial cancer in the TCGA database, divided into high immunity and low immunity groups. A total of 721 differentially expressed genes were screened, including 633 upregulated genes and 88 downregulated genes. According to go and KEGG analysis of differentially expressed genes, upregulated DEGs were mainly enriched in the allograft, complement system, inflammatory mediators, IFN-*α*, IFN-*γ*, and other signalling pathways, while downregulated DEGs were primarily enriched in E2F, mitotic, G2M, and different signalling pathways. The key genes were VEGFA, CCL2, and IFN genes. In univariate independent prognostic analysis, the risk score was *P* < 0.05, indicating that the risk score can be used as an independent prognostic molecule. The results suggest that VEGFA, CCL2, and IFN genes may be the critical gene targets in endometrial carcinoma.

The article "Construction of an Immune-Autophagy Prognostic Model Based on ssGSEA Immune Scoring Algorithm Analysis and Prognostic Value Exploration of the Immune-Autophagy Gene in Endometrial Carcinoma (EC) Based on Bioinformatics" was retracted in 2023. Reasons: signs of a paper mill; suspected computer-generated content; unreliable results or conclusions; concerns about the data.

There are six secretion subtypes in the VEGF family: VEGF-A, VEGF-B, VEGF-C, VEGF-D, VEGF-E, and placental growth factor [33]. VEGF-A is an endothelial cell-specific growth factor regulating angiogenesis. It is an effective stimulator in angiogenesis and is involved in multiple tumour types, including endometrial carcinoma [34]. lncRNA-TDRG1 may promote endometrial cancer's occurrence and regulate VEGF-A downstream protein expression [35, 36]. Mir-140-5p can reduce ovarian cancer angiogenesis and inhibit cancer progression by downregulating VEGFA expression. The mir-140-5p can reduce ovarian cancer angiogenesis and inhibit cancer progression by downregulating VEGFA expression. More than 50% of tumours overexpress VEGF-A in endometrial carcinoma and have a poor prognosis [37]. The high expression of VEGF and VEGFR in preoperative serum is closely related to angiogenesis and malignant phenotype and is a prognostic factor of endometrial cancer [38, 39].

Inflammatory factors generally involve inflammatory chemokines, especially CCL2 is related to tumour progression. CC chemokine ligand 2 (CCL2) belongs to the chemokine CC family, can raise tumour-related macrophages, promote tumour angiogenesis, and regulate the immune response. The expression level of ccl2mrna in breast cancer tissue is 13.18 times higher than in adjacent tissues [40]. A high level of CCL2 is positively correlated with TNM stage and lymph node metastasis of gastric cancer [41]. CCL2 may be involved in the invasive growth of gastric cancer. The high level of CCL2 expression in gastric cancer indicates a poor prognosis of gastric cancer. In the study of endometrial cancer, the inactivation of LKB1 leads to the abnormal expression of inflammatory cytokine chemokine in the tumour, leading to the increase of macrophage recruitment with significant tumour-promoting activity [42]. The study showed that CCL2 expression is an important prognostic factor of cancer [43].

IFNs (interferons) are a group of signalling proteins synthesized and released by host cells in response to pathogens. Under normal circumstances, the virus-infected cells will release interferon, making the surrounding cells improve their antivirus defence ability. Based on the receptor type, human interferon can be divided into three types: type I interferon, including IFN-*α*, IFN-*β*, type II interferon (known as IFN-*γ* in humans), and type III interferon. In many tumour studies, IFN-*α* and IFN-*β* can promote and inhibit tumour cells, which may be an important prognostic factor of cancer. The connection between IL-18 and its receptor activates the MyD88 signalling pathway, inducing IFN-*γ* production. In terms of the tumour, tumour-infiltrating lymphocytes (TIL) are the primary source of IFN-*γ*, which has shown special significance in tumour immune monitoring [44]. Studies have shown that IFN-*γ* has dual effects on tumour cells.

The article "Construction of an Immune-Autophagy Prognostic Model Based on ssGSEA Immune Scoring Algorithm Analysis and Prognostic Value Exploration of the Immune-Autophagy Gene in Endometrial Carcinoma (EC) Based on Bioinformatics" was retracted in 2023. Reasons: signs of a paper mill; suspected computer-generated content; unreliable results or conclusions; concerns about the data.

On the one hand, IFN-*γ* can inhibit the growth of human melanoma cells in vitro. On the other hand, it can increase HLA-DR expression and other tumour markers in advanced melanoma. It indicates that IFN-*γ* may promote the development of more aggressive phenotypes in cancer cells. Relevant studies have shown that IFN-*γ* can promote tumour occurrence and then promote the change of tumour cell phenotype to improve the growth adaptability of the immuno-competent host [45]. Studies have shown that interferon-*α* (IFN-*α*) downregulates the expression of cyclooxygenase-2 in bladder cancer cells by inhibiting the tpl2/NF-*κ*B pathway. IFN-*α* also inhibits the COX-2 expression by inhibiting cAMP signal transduction of PDE4D activity mediated by tpl2-erk. PDE4D can enhance the antitumour effect of IFN-*α* on bladder cancer [46]. Meanwhile, studies found that differential expressed genes may be one of the reasons for the different drug sensitivity in patients with the related disease. Therefore, this study predicted four potential therapeutic drugs sildenafil, sunitinib, TPCA-1, and etoposide to provide certain drugs support for clinical treatments of endometrial cancer, which may work through differential expression of genes [47]. In addition, autophagy is an intracellular self-degradative process providing elimination of damaged or dysfunctional organelles under stressful conditions such as nutrient deficiency, hypoxia, or chemotherapy. Interestingly, the signalling pathways that are involved in cancer-associated inflammation may regulate autophagy as well [48, 49].

### 3.1. Limitations

This study is based on bioinformatics methods and uses various tools and software to process and analyze a large number of data. However, there are still shortcomings: (1) first, the predicted prognostic genes should be further verified to observe their specific role in vitro in EC. (2) Secondly, experimental data should be used to verify the stability and accuracy of the prognosis model. (3) Finally, experimental evidence should be used to study further the effects of potential drugs predicted by Camp and CTRP 2.0 on EC treatment. In future research, we hope to collect our own experimental and clinical data, further explore the mechanism of molecular biology level, build a more reliable and stable prognosis prediction model, and apply this model to clinical, which can better serve patients.

The article "Construction of an Immune-Autophagy Prognostic Model Based on ssGSEA Immune Scoring Algorithm Analysis and Prognostic Value Exploration of the Immune-Autophagy Gene in Endometrial Carcinoma (EC) Based on Bioinformatics" was retracted in 2023. Reasons: signs of a paper mill; suspected computer-generated content; unreliable results or conclusions; concerns about the data.

## 4. Conclusion

In summary, this study constructed a prognostic model of endometrial cancer based on 22 immune-related genes by mining TCGA and HADB databases. Finally, it identified three high-risk genes as prognostic genes of endometrial cancer, including VEGFA, CCL2, and IFN. The identification of these genes will also provide new possibilities for the treatment and intervention of endometrial cancer. At the same time, the drug sensitivity test showed that four potential therapeutic drugs were sildenafil, sunitinib, TPCA-1, and etoposide, to provide certain drugs support for the treatment of endometrial cancer.

## Figures and Tables

**Figure 1:** Development and validation of two immune cell subtypes in EC TCGA cohort. (a) When *k* = 2, the consensus score matrix of the EC sample is higher. The higher consensus score between the two samples indicates that they are more likely to be assigned to the same cluster in different iterations; (b) EC described the real random variables of its probability distribution, based on the consensus scores of different subtype numbers (*k* = 2–10); (c) the trigonometric curve of all samples is *k* = 2; (d) CTLA-4 was differentially expressed in the two subtypes; (e) the differential expression of CD274 in the two subtypes was observed; (f) the expression of PDCD1 was different between the two subtypes; (g) ssGSEA fractional thermogram of 28 kinds of immune cells.

**Figure 2:** Difference analysis of DEGs genes. (a) Immunity_H and Immunity_L Kaplan–Meier curve; (b) differential distribution heat map of 721 DEGs genes; (c) volcano map of differential gene expression; red represents upregulation; green represents downregulation.

**Figure 3:** Go and KEGG enrichment analysis and immune infiltration analysis; (a) KEGG enrichment analysis of upregulated DEGs; (b) KEGG enrichment analysis of downregulated DEGs; (c) Go enrichment analysis of DEGs; (d) heat map of immune infiltration correlation.

**Figure 4:** Construction and evaluation of prognostic model; (a) Venn diagram map of DEGs, autophagy, and immune genes; (b) risk curve of endometrial cancer patients; (c) univariate Cox independent prognostic analysis; (d) risk classification test heat map.

The article "Construction of an Immune-Autophagy Prognostic Model Based on ssGSEA Immune Scoring Algorithm Analysis and Prognostic Value Exploration of the Immune-Autophagy Gene in Endometrial Carcinoma (EC) Based on Bioinformatics" was retracted in 2023. Reasons: signs of a paper mill; suspected computer-generated content; unreliable results or conclusions; concerns about the data.

**Figure 5:** Drug sensitivity test: (a) drug Venn diagram; (b-c) Spearman correlation analysis and drug response difference analysis results.

## Data Availability

The data used to support this study are available from the corresponding author upon request.
